# Path Realization and Analysis of Synergy between Ecological Environment Development and Innovative Entrepreneurship Education

This article has been retracted.

**DOI:** 10.1155/2022/8634134

**Published:** 2022-08-23

**Authors:** Zikang Peng

**Affiliations:** School of Marxism, Henan Finance University, Zhengzhou, Henan 450046, China

## Abstract

In the context of implementing an innovation-oriented development strategy in China, innovation and entrepreneurship education in colleges and universities has increasingly become the focus of government and society. Entrepreneurship education is a complex ecosystem, which includes the collaboration among universities, government, and enterprises as well as the effective integration of educational resources inside and outside the university. How to establish a new type of government, universities, and enterprises to jointly cultivate innovative talents is a major issue that universities in China urgently need to solve at present. This study tries to provide some useful insights for innovation and entrepreneurship education in China's colleges and universities, starting from the development of the ecosystem and the cooperation model in the teaching of innovation and entrepreneurship education.

## 1. Introduction

Joseph Schumpeter's Theory of Economic Development states that “innovation is the most important driver of economic growth” [1]. As shown in Figure 1 Bear-Peter's innovation. Innovation requires innovation education to produce a large number of innovative people. By educating students, innovation education enables them to accept and discover new ideas, new knowledge, new methods and new things, to grasp the laws contained therein, to develop their individual creative spirit and innovative abilities, and to lay the quality foundation for continuous innovation. The implementation of innovation education cannot be achieved without a good educational ecological environment, of course, a bad ecological environment is counter-productive to the effectiveness of innovation education. The educational ecological environment covers all aspects of nature and society in the field of education, including the natural environment social environment, school environment, network environment, and other internal and external influencing factors. Innovative talents should have the courage to explore unknown fields, the innovative spirit to pursue truth, meticulous thinking and vigorous energy, and be complex talents who are proficient in specific fields of expertise or have a wide range of disciplines. “It takes ten years to grow a tree but a hundred years to nurture a man” [2]. In the process of nurturing people, a good educational and cultural ecological environment helps students develop physically and mentally and cultivate innovative qualities. Therefore, it is of great practical significance to build an ecological development environment that is holistic, harmonious, interactive and symbiotic, and open to development.

As shown in Figure 2, the data from 2016–2020 show that many foreign scholars have conducted research on “innovation and entrepreneurship education.” The research results tend to be at a stable level, which indicates that the research on “innovation and entrepreneurship education” has received a lot of attention abroad.

As shown in Table 1, eco-entrepreneurship, also known as green entrepreneurship, environmental entrepreneurship, low carbon entrepreneurship, and sustainable entrepreneurship, was first proposed by Professor Quinn. As an emerging research topic in the field of entrepreneurship, the terminology of green entrepreneurship has not been uniformly defined, with most researchers using the term “green entrepreneurship,” and some researchers in the English literature also using “environment In the English literature, some researchers also use the terms “environmental entrepreneurship,” “ecopreneurship” and “sustainopreneurship” to describe it, while the definition of green entrepreneurship has not yet been standardized. The definition of green entrepreneurship has not yet been standardised [3].

Ecology is the macro-biology that studies the patterns of interaction between individuals, populations, or communities of organisms and their environment and their mechanisms [4]. Ecology is concerned with ecosystems and ecological balance. An ecosystem is a unified whole in which all organisms (including individuals, populations, and communities) in a given territory or space interact with each other and with their inorganic environment, emphasizing the interconnectedness, interdependence, and interconnection of all factors in the system [5]. As society is a complex system, many of the activities of human society are modeled on natural ecosystems, so the research perspective and methods of ecology are gradually being extended from the natural sciences to the social sciences. The birth of the emerging discipline of educational ecology is the result of the application of ecological principles, laws, and methods in the field of education [6]. The expansion of ecological niches can further contribute to the sustainable development of a particular species. This thesis intends to analyze the innovation and entrepreneurship education ecosystem and its internal and external environment, and discuss it in detail from the perspective of “three-dimensional linkage” of cultural environment, resource environment, and institutional environment.

## 2. State of the Art

### 2.1. Domestic Development Status

It has only been more than ten years since the “Tsinghua University Entrepreneurial Plan Competition” started in 1997. In 1999, the Action Plan for Revitalization of Education in the 21st Century proposed to “increase the efforts to encourage teachers and students to start their own high-tech companies” and launched the Challenge Cup Student Entrepreneurship Competition. As shown in Figure 3, In 2002, a pilot project of entrepreneurship education was launched in some universities. In recent years, an entrepreneurial spirit has emerged in universities. In the current pilot entrepreneurship education programs, the Bureau of Entrepreneurship Education is limited to imparting knowledge and lacks sufficient space for practice and development, and is not integrated with the overall education system of the university. Entrepreneurship education is not “formal education,” but a kind of “non-formal education” which is engaged in “amateur education” in spare time, and it can even be said to be “Therefore, entrepreneurship education is only superficial, not deep, and not really “spiritual”.

In the late 1960s, based on the important impact of entrepreneurial entrepreneurs on the economic and social structure of the United States and the world, a group of outstanding economists from the Bacon-School of Business, represented by Professor Timmons, predicted that “the United States was in the midst of a quiet revolution.” This is the first time a new model of entrepreneurship education has been proposed.

### 2.2. Analysis of the Synergy Problem of Innovation and Entrepreneurship Education in the Ecosystem

After more than two decades of development, innovation and entrepreneurship education have begun to bear fruit, and the scale and number of various types of college students' entrepreneurship parks and entrepreneurial enterprises have been expanding, the proportion of college students participating in entrepreneurship has been increasing, and the success rate of entrepreneurship has been rising [7]. However, compared with the innovation and entrepreneurship education in foreign universities, there is still a certain gap. The cooperative cultivation of students and students in colleges and universities is a complex ecological system, and each collaborative cultivation subject has different degrees of problems in this system.

1. The lack of interaction between the collaborative training subjects in innovation and entrepreneurship education has a great impact on its teaching quality [8]. At present, the innovation and entrepreneurship education of college students in government-school, school, enterprise, and government-enterprise shows a lack of collaborative development and the effect of cooperation is not significant. As shown in Figure 4, The main manifestations are as follows: First, the cooperation between government and school. At present, the cooperation between universities and local governments in China is not strong, the advantages of universities in terms of professional and human resources are not fully reflected, and most local governments do not stand on the height of providing innovative talents for local economic development. The policy of innovation and entrepreneurship education for college students should be forward-looking, which somehow restricts the innovation and entrepreneurship ability of college students. Second, at the level of cooperation between enterprises and universities, the connection between universities and companies is still very weak. The main manifestations are: first, a “win-win” cooperation model has not been formed between universities and enterprises. As a practical place to test the effectiveness of university students' innovation and entrepreneurship education, enterprise is also a key link from “innovation” to “innovation and entrepreneurship” in universities. However, due to the disconnection between theory and practice, its “supply” cannot be adapted to the “demand” of enterprises. At the level of cooperation between the state and enterprises, it is mainly reflected in the lack of cooperation mechanism between the state and enterprises with innovation and entrepreneurship education as the core. The synergistic cultivation effect formed by the linkage between the state and enterprises is greatly weakened, and the innovation and entrepreneurship services provided by enterprises for universities, such as establishing various practice platforms, are not sufficiently supported by the state, and enterprises are not highly motivated to promote innovation and entrepreneurship education.
2. A fragmentary understanding of the concept of implementation [9]. Two ways of thinking to promote the development of innovation and entrepreneurship education for college students are: ecological and elemental [10]. The ecological mode of thinking advocates the holistic nature of education and the balance and interaction in the innovation and entrepreneurship education system. The “elemental” mode of thinking, on the other hand, advocates “partial-centeredness” and focuses on the connection between “partial” and “whole.” The “elemental” mindset advocates a “part-centered” approach, focusing on the connection between “part” and “whole.” The “elemental” mode of thinking advocates a “part-centered” approach, focusing on the connection between the “part” and the “whole.” The elementalized teaching model can quickly find a way out of the current innovation and entrepreneurship education, but its internal logic is fractured and is likely to lead to problems later on. Therefore, the current universities must correctly understand the core idea of innovation and entrepreneurship education, deeply understand the connotation of innovation and entrepreneurship education, and understand the relationship between its connotations. At present, colleges and universities should correctly understand the core idea of innovation and entrepreneurship education, deeply understand the connotation of innovation and entrepreneurship education, and understand the relationship between its connotation, which is an important part of building innovative education. In terms of national policy, “innovation and entrepreneurship education” was proposed by the Ministry of Education in 2010 as a way to promote social and economic development. Many scholars have analyzed the reasons for its creation in order to deepen their understanding. At present, there is a consensus among universities that innovation and entrepreneurship education should be aimed at improving the overall quality of college students. However, as far as the current actual situation is concerned, there are some misconceptions among students, teachers, schools, and even the society and government that entrepreneurship is a matter for a few people and poor students.
3. The superficiality of the implementation results is embedded [11]. As shown in Figure 5, The factors in the innovation and entrepreneurship ecology are interdependent and cannot constitute a complete cycle without a single link. In the vision of education ecology, the establishment of an innovation and entrepreneurship education community is not the superposition of each factor, but the organic combination of each factor. To promote innovation and entrepreneurship education for college students, it cannot be placed within the original university education system. First, it is difficult to combine vocational education and innovation and entrepreneurship education, therefore, all universities have to seriously consider how to integrate innovation and entrepreneurship education into vocational education, which requires the overall quality of teachers [12]. Second, there is a conflict between the existing university education system and the new innovation and entrepreneurship education, and the traditional teaching model is too rigid to adapt to the actual needs of enterprises. Third, the subjective initiative of the participating subjects is not enough, resulting in the entrepreneurial spirit of the whole enterprise has not yet been formed.

## 3. Methodology

### 3.1. Exploring the Path of Innovation and Entrepreneurship Education in Universities under the Ecological Perspective

The establishment of a sound talent cultivation mechanism for college students' innovation and entrepreneurship education is explored. Focus on several aspects such as teaching team, teaching system, service support platform, innovation and entrepreneurship culture atmosphere, innovation and entrepreneurship environment, and innovation and entrepreneurship evaluation system.

First, the construction of the teaching staff should broaden the channels of introducing teachers as far as possible, combine introduction and cultivation with the practical situation of our university, and actively introduce tutors with an industrial background outside the university, such as senior managers of enterprises with rich practical experience, etc. We can also encourage young teachers of our university to enter enterprises for practice, so as to ensure that professional teachers have a high level of practical knowledge, whether in theoretical lectures or practical links, and can combine with the current industrial development The second is to build a sound teaching system.

Second, a perfect teaching system is constructed [13]. In the whole process of entrepreneurship education, entrepreneurship education should be carried out at every stage and at different stages of education. At the basic education level, the main purpose is to cultivate students' innovation consciousness, while at the higher education level, the main purpose is to enhance students' innovation consciousness and improve their innovation ability. The main purpose of “liberal” initiation education is to foster entrepreneurship, entrepreneurial awareness, independent work, and continuous learning. In order to achieve the goal of universal enlightenment, to connect the chain of entrepreneurship education in schools, and to prevent the lack of school education, it is necessary to strengthen entrepreneurship education at the basic education level.

Third, we should build a support platform for innovation and entrepreneurship education in colleges and universities. On the one hand, we should improve the internal management service system of colleges and universities, coordinate the connection of various departments and faculties of colleges and universities, provide professional and high-level services for innovation and entrepreneurship, and form a good social atmosphere in which colleges and departments of colleges and universities actively support innovation and entrepreneurship. In addition, it can also create a better employment environment for college students and provide a perfect guarantee for innovation and entrepreneurship education.

Fourth, we set up associations for college students, such as “Ecological Protection Association,” “Ecological Entrepreneurship Association,” “Ecological Entrepreneurship Association,” “Ecological Entrepreneurship Competition “The association will carry out activities such as “ecological entrepreneurship competition” and “ecological design competition” in order to stimulate the “inner motivation” of college students. The purpose is to stimulate the “intrinsic motivation” of college students through the activities of clubs such as “eco-entrepreneurship competition” and “eco-design competition.” Fifth, we should build a platform for school-enterprise cooperation. Universities should give full play to their disciplinary and professional advantages, rely on the high-tech parks in the park and the ecological resources of the park, promote school-enterprise cooperation and the combination of production, learning and research, and build a comprehensive ecological internship base, as shown in Figure 6.

“Personality education reform” is implemented to stimulate the sustainable development of talents. Personality is the source of innovative spirit, and innovative education must be based on personality education. In order to equip students with the motivation for innovation and sustainable development, universities should do a good job of “personality education reform”.

A good ecological environment is created for enterprises [14]. Integrating ecological entrepreneurship education into campus culture construction can play a long-term and profound role in the ideological behavior of college students, as well as effectively promote the cultivation of entrepreneurial consciousness and the quality of entrepreneurship among college students [15]. Industrial civilization, driven by modern technology, has promoted a leap in productivity, but it has also gradually severed the link between human beings and nature. Humans began to move toward the opposite side of nature, and the destruction of ecosystems expanded rapidly, eventually triggering a global ecological crisis. How to cope with the deteriorating ecological environment and how to ensure the sustainable development of human society is a major challenge for human beings and an important issue for education reform [16]. Adhering to the ecological concept is the biggest difference between ecological entrepreneurship and traditional entrepreneurship, and this concept is reflected in three changes: the concept of “conquering nature” is changed to the concept of “harmony between man and nature”; the growth mode of excessive consumption of resources is changed to the growth mode of sustainable development; the development mode of emphasizing material things rather than people is changed. The growth model of excessive consumption of resources is changed to the growth model of sustainable development; the development concept of emphasizing things over people is changed to the development concept with the overall development of people as the core [17]. The concept of ecology is integrated into innovation and entrepreneurship education, which is the echo of education to the construction of ecological civilization.

Depending on their educational goals, they can be divided into two categories: centralized and decentralized, as shown in Table 2.

### 3.2. The Realization Path of Constructing Ecological Innovation and Entreprene-Urship Education

Eco-environmental education provides the basis for college students to start their own businesses. To improve the quality of eco-entrepreneurship education, a corresponding curriculum system needs to be constructed [18]. Universities should integrate the concept of green, low-carbon, and coordinated ecological development into their overall teaching planning, realize the organic integration of ecological entrepreneurship content with the professional curriculum system, professional practical teaching, and ecological entrepreneurial activities, and explore ecological innovation and entrepreneurship education methods that fit with professional education. Ecological education is the foundation of eco-entrepreneurship among university students. Upholding the concept of ecological development, exploring the construction of a teaching and practice system for eco-entrepreneurship education for university students from the aspects of the education concept, target orientation, curriculum, practice platform, resource guarantee, and atmosphere formation is an important task for innovation and entrepreneurship education in universities.

As shown in Figure 7, the “time lag effect” in the narrow sense of “entrepreneurship” requires attention to endogenous and exogenous factors that influence entrepreneurial intention and behavior. Create a practical platform for ecological entrepreneurship education [19]. Practice is an effective way to strengthen entrepreneurship education for university students. On the basis of constructing a curriculum system related to ecological entrepreneurship education, universities must integrate resources from inside and outside the university and focus on creating “five platforms”: First is an experimental training platform, encouraging teachers to introduce entrepreneurial projects in line with the direction of ecological development into the laboratory or virtual experimental platform, so that students can practice and experience them according to the requirements of teaching and training. Second is a platform for scientific and technological competitions, based on ecological concepts and around ecological themes, to create various competitions based on high-level competitions such as “Internet+” and “Challenge Cup” to cultivate students' ecological thinking and encourage them to put ecological entrepreneurship into practice. Third is a platform for practice and incubation. Colleges and universities should consciously and keenly put in and introduce ecological projects for students to practice and incubate through crowdsourcing spaces and university student business parks. The fourth is the platform of student associations, giving full play to the role of student associations, forming associations such as the Ecological Protection Association and the Ecological Innovation and Entrepreneurship Association, and organizing a series of association activities such as the Ecological Entrepreneurship Plan Competition and the Ecological Theme Design Competition to stimulate the inner motivation of students. Fifth, to build a school-enterprise cooperation platform, the use of local high-tech industrial parks, parks resources, school-enterprise cooperation, industry-university-research combination of comprehensive practice base.

Create an ecological entrepreneurial culture [20]. Incorporating eco-entrepreneurship education into the construction of campus culture can have a lasting and deep impact on students' thinking and behavior, and can effectively stimulate their entrepreneurial consciousness and cultivate their entrepreneurial psychological qualities.

As shown in Table 3, in simple terms, a consumer in nature is a group of organisms that can only survive by consuming other organisms without being able to produce themselves. As consumers, local universities and local enterprises play an important role as the driving force in the on-campus support system for innovation and entrepreneurship education. It is necessary to organically combine the needs of the times of ecological civilization and the creativity of college students, to take the construction of ecological civilization as an important content of talent training, and to truly integrate the concept of ecological development into the concept of nurturing people in universities through continuous reform and improvement in order to cultivate ecological innovative and entrepreneurial talents who meet the requirements of the times. Eco-entrepreneurial culture is a broad concept, covering the value system, ideology, and psychological awareness formed by university students in the process of creating values and realizing the harmonious coexistence between human beings and nature, which has a direct impact on their behavior and way of thinking.

## 4. Result Analysis and Discussion

### 4.1. Analysis of the Composition of Innovative Entrepreneurship Education Ecosystem

The essence of a disciplinary innovation ecosystem is a collaborative integration among organizations [21], integrating the innovative products of core disciplines and relevant partner organizations along the value chain from initiation to implementation and from successful innovation to the realisation of value to form a coherent, demand-oriented solution. Based on the literature research, the disciplinary innovation ecosystem is divided into three levels from inside to outside in the order of core, collaborative, and value realization layers according to the whole process of disciplinary innovation activities carried out.

As shown in Figure 8, the core tier is the disciplinary innovation platform, where the core disciplines gather various forces to establish the best combination of capabilities, talents, processes, technologies, research systems, and funding for potential needs, in order to provide the new value space needed for potential needs, and is the key force to ensure the successful implementation of disciplinary innovation. In the collaborative layer, technical support providers, competing disciplines, technical standard recognition bodies, strategic partners, and core disciplines interact through knowledge chains, competitive cooperation, or other internal linkage models, while various nutrition providers (infrastructure providers, industry associations, technical service agencies, and other service organizations) provide intellectual support for disciplinary innovation in terms of knowledge flow, technology flow, human resource flow, information flow, and other production factors support. After the successful implementation of disciplinary innovation, the most important link is the promotion of the innovation results [22]. The value realization layer plays a very important role in the diffusion of disciplinary innovation. The promoters of innovation results according to the needs of different levels and the trend of demand in order to further explore the potential demand; the government influences disciplinary innovation through the innovation policy system, and the actors of core disciplinary innovation make full use of government policies to give a macro and systematic perspective to The government influences disciplinary innovation through its innovation policy system.

### 4.2. Analysis of Knowledge Innovation Mechanism of Innovation and Entrepreneurship Education Ecosystem

A discipline is a specialized and organized collection of knowledge and competencies, and any innovation can be seen as a process of generating new knowledge [23]. The three stages of knowledge innovation in a disciplinary innovation ecosystem are the process of continuously adjusting its knowledge structure according to the changes in environmental factors and carrying out knowledge inheritance under the joint action of the knowledge storage mechanism, the knowledge circulation mechanism, and the knowledge integration mechanism. These three mechanisms together constitute the knowledge innovation mechanism of the disciplinary innovation ecosystem, and the three are inextricably linked and influenced by each other. Knowledge storage provides knowledge resources to support knowledge innovation, and through knowledge circulation within the system, each member obtains learning resources, and finally, through knowledge integration, knowledge innovation within the system is successfully implemented. Under the synergy of the three mechanisms, from knowledge storage, to knowledge circulation, and then to knowledge integration, after achieving the qualitative change of knowledge innovation in the disciplinary innovation ecosystem, a new cycle will start because of the introduction of new knowledge, and the knowledge innovation within the discipline is always in a dynamic cycle state of continuous self-renewal, which is finally reflected in the continuous enhancement of the core competitiveness of the discipline, as shown in Figure 9.

The knowledge innovation mechanism of the innovation and entrepreneurship education ecosystem should embody the university, industry, and government while retaining their original roles and unique identities, each exhibiting some other two capabilities. The three parties are cooperative and their roles are interchanged.

## 5. Conclusion

To sum up, educational ecology is a kind of educational research perspective and method to analyze the current situation of education and promote the development of education. By using the principles of ecology to analyze and solve educational problems, it reveals the mechanism and laws of ecological development of education. This study investigates innovation and entrepreneurship education based on the research perspective of educational ecology and proposes targeted strategies to promote the ecological development of innovation and entrepreneurship education in response to the problems existing in the current development of innovation and entrepreneurship education, which is considered to have certain research significance and value for the development of innovation and entrepreneurship education.

In conclusion, as a new form of education that responds to the development of the times and has a positive impact on all aspects of society, politics, economy and culture, entrepreneurship education, although it started relatively late in China, it has made some achievements and shown a trend of flourishing due to the attention and support from the government and all walks of life. In this background, colleges and universities should start from the actual needs of college students, combine the advantageous resources of schools, actively explore and study the ways and methods of entrepreneurship education, and establish the entrepreneurship education ecosystem of enterprises from the intrinsic factors of enterprises, build a multi-level and diversified practice platform, and promote the sustainable development of entrepreneurship education ecosystem based on the integration of practice and practice.

## Figures and Tables

**Figure 1:** Bear-Peter's innovation.

**Figure 2:** Trends in the number of relevant publications in foreign countries in the past five years.

**Figure 3:** The planning of job creation in China and innovation-driven economies.

**Figure 4:** Ecological network model of government, school, and enterprise.

**Figure 5:** Ecological framework of innovation and entrepreneurship.

**Figure 6:** Cognitive map of creativity and inventiveness of students in higher education.

**Figure 7:** The “time lag effect” of innovative entrepreneurship education.

**Figure 8:** Composition of the disciplinary innovation ecosystem.

**Figure 9:** Knowledge innovation mechanism of disciplinary innovation ecosystem.

**Table 1:** definition of eco-entrepreneurship.

Scholars	Definition
Dean&McMullen “entrepreneurial opportunism”	The process of identifying, evaluating, and exploiting business opportunities that arise from market failures and are closely related to the environment, based on the goal of sustainable development
Cohen&Winn	Focus on opportunities to bring the goods and services of the “future” to life and leverage innovation capabilities and the ability to identify and analyze opportunities to develop new green markets
Nelson&Sumesh	Tendency to create and innovate “green” organisations, making green resources the core competence of enterprises to develop green markets
Schape	Demonstrate advanced management concepts and business strategies to guide enterprises to be more proactive in achieving economic benefits through greening

**Table 2:** Classification table of innovation and entrepreneurship education model.

Model classification	Refinement model	Important conditions to rely on
Focused	Research project incubation model	Research project incubation model
	Government-industry-academia-research-application cooperation model	Government actions support; financial institutions support

Dispersed	Professional practice model	Enterprise platform; simulation platform
	Integrated model	Top-down top-level design

**Table 3:** Table of elements of the ecosystem of in-school support system for innovation and entrepreneurship education.

Roles	Corresponding elements	Role
Producers	Course system and faculty	Innovation and entrepreneurship creativity and innovation and entrepreneurship education theory
Decomposer	Supporting organisations on campus	Innovation and entrepreneurship education and practice technology, information and consulting services
Environment	Policy system and cultural environment	Institutional guarantee of innovation and entrepreneurship and cultural atmosphere of entrepreneurship education

## Data Availability

The labeled dataset used to support the findings of this study is available from the corresponding author upon request.
